# siRNA-mediated knockdown against NUF2 suppresses pancreatic cancer proliferation *in vitro* and *in vivo*

This article has been retracted.

**DOI:** 10.1042/BSR20140124

**Published:** 2015-01-14

**Authors:** Peng Hu, Xi Chen, Jing Sun, Ping Bie, Lei-Da Zhang

**Affiliations:** *Department of Hepatobiliary Surgery, Southwest Hospital, Third Military Medical University, ChongQing, China

**Keywords:** NUF2, pancreatic cancer, RNA interference, tumourigenesis, treatment, *C*_T_, threshold cycle value, GAPDH, glyceraldehyde-3-phosphate dehydrogenase, HEK, human embryonic kidney, HRP, horseradish peroxidase, MTT, 3-(4,5-dimethylthiazol-2-yl)-2,5-diphenyl-2*H*-tetrazolium bromide, PCNA, proliferating cell nuclear antigen, PDAC, pancreatic ductal adenocarcinoma, RNAi, RNA interference, RT–PCR, reverse transcription–PCR, shRNA, small hairpin RNA, siRNA, small interfering RNA

## Abstract

NUF2 (NUF2, Ndc80 kinetochore complex component) plays an important role in kinetochore-microtubule attachment. It has been reported that NUF2 is associated with multiple human cancers. However, the functional role of NUF2 in pancreatic cancer remains unclear. In this study, we found that NUF2 expression was stronger in tumour tissues than in normal pancreatic tissues, and its overexpression could be related to poor prognosis. Moreover, NUF2 was highly expressed in several human pancreatic cancer cell lines. We took advantage of lentivirus-mediated siRNA (small interfering RNA) to suppress NUF2 expression in PANC-1 and Sw1990 cell lines aiming to investigate the role of NUF2 in pancreatic cancer. NUF2 silencing by RANi (RNA interference) reduced the proliferation and colony formation ability of pancreatic cancer cells *in vitro*. Cell cycle analysis showed that NUF2 knockdown induced cell cycle arrest at G0/G1 phase via suppression of Cyclin B1, Cdc2 and Cdc25A. More importantly, NUF2 silencing was able to alleviate *in vivo* tumourigenesis in pancreatic cancer xenograft nude mice. Collectively, the present study indicates that the siRNA-mediated knockdown against NUF2 may be a promising therapeutic method for the treatment of pancreatic cancer.

## Abstract 2

NUF2 is overexpressed in pancreatic cancer tissues and cell lines. siRNA-mediated knockdown against NUF2 resulted in a significant reduction in pancreatic cancer cell growth both *in vitro* and *in vivo*. NUF2 may be a promising therapeutic target in pancreatic cancer.

## INTRODUCTION

Pancreatic cancer is one of the most lethal human cancers worldwide with a mortality rate in excess of 95% of its incidence rate [1,2]. Surgical resection such as pancreaticoduodenectomy is suitable for patients with localized pancreatic cancers [3], but is only appropriate for up to 15–20% of patients [4]. Approximately 80% of pancreatic cancers are either locally advanced or metastatic upon diagnosis, which show a high aggressive nature invading mainly regional lymph nodes and liver [5]. In the last two decades, strategies, including surgery, radiation and chemotherapy, have failed to improve long-term survival [6]. The current standard of treatment for unresectable or metastatic pancreatic cancer, the nucleoside analogue Gemcitabine, however, prolongs survival by only several months [7]. Therefore innovative diagnostic and therapeutic strategies are urgently required nowadays.

To maintain the genomic integrity, proper and accurate chromosome segregation is necessary, which requires an appropriate coordination among chromosomes, kinetochores and spindles during mitosis. The kinetochore is a large, multi-protein structure that is assembled at the centromere of each sister chromatid pair in mitosis. The kinetochore has an inner core containing the CENP-A, CENP-B and CENP-C proteins that anchor the kinetochore to centromeric DNA [8], and outer domains containing spindle checkpoint proteins Mps1, Mad1, Mad2, Bub1, BubR1, Bub3, Cdc20, microtubule-interacting proteins EB1, APC, Clip170, Clasp1, and motor proteins, including Cenp-E, dynein [9]. Besides, its middle domains contain two heterodimers of Ndc80-NUF2 and Spc24-Spc25, which have been suggested to be necessary in formation of stable microtubule–kinetochore attachment, chromosome alignment, and spindle checkpoint activation in mitosis [10]. NUF2 (NUF2, Ndc80 kinetochore complex component), also named as CDCA1 (cell division associated 1), is part of a molecular linker between the kinetochore attachment site and tubulin subunits within the lattice of the attached plus ends [11]. DeLuca *et al*. found that in HeLa cells, after knockdown of NUF2 by RNAi (RNA interference), spindle formation occurred normally, but kinetochores failed to attach to spindle microtubules and cells block in prometaphase, which caused aberrant chromosome segmentation and induced mitotic cells to undergo cell death [12]. Dysregulation of Ndc80-NUF2 has been employed in the development of a series of human cancers, including lung cancer, colorectal cancer, gastric cancer, prostate cancer, urinary bladder cancer, renal carcinoma and ovarian cancer, rather than other normal tissues except testis [13–18]. It has been found that depletion of NUF2 by specific siRNAs (small interfering RNAs) resulted in inhibition of cell proliferation and induction of apoptosis in non-small-cell carcinoma and ovarian cancer [17,18]. Likewise, in colorectal and gastric cancers, after the siRNA-mediated knockdown against NUF2, cell growths were significantly suppressed, and subG1 fractions of cell cycle were significantly increased [15]. Furthermore, NUF2 was found be significantly related to the risk of prostate cancer recurrence following radical prostatectomy [13]. Recently, high level of NUF2 expression was reported to be associated with poor prognosis for patients with colorectal cancers [19]. Together, these results highlight a specific role of NUF2 in tumour growth and metastasis and make it a potential candidate for molecule-targeted therapy in many cancers.

In the present study, we found that NUF2 is highly expressed in human pancreatic cancer specimens rather than adjacent non-cancerous tissues. Moreover, NUF2 is extensively expressed in several human pancreatic cancer cell lines. Thus we used lentivirus-mediated siRNA targeting NUF2 to suppress its endogenous expression in pancreatic cancer cells with the aim of examining the role of NUF2 in pancreatic cancer and developing a novel therapeutic strategy for pancreatic cancer. To the best of our knowledge, it is the first report to investigate the function of NUF2 in the development of pancreatic cancer.

## MATERIALS AND METHODS

### Cell culture

Human pancreatic cancer cell lines Sw1990, PANC-1, BXPC-3 and MLA-PACA-2 and HEK (human embryonic kidney) 293 cells were obtained from the Cell Bank of Chinese Academy of Sciences (Shanghai, China), and cultured in DMEM (Dulbecco's modified eagle's medium) (Hyclone) containing 10% (v/v) FBS (Biowest), 100 units/ml penicillin and 100 mg/ml streptomycin (Hyclone). All cell lines were maintained in a humidified atmosphere of 5% (v/v) CO_2_/air at 37°C.

### Immunohistochemistry

In our study, tumour specimens from 128 patients who underwent surgery for PDAC (pancreatic ductal adenocarcinoma) from 2006 to 2012 at Southwest Hospital (Chongqin, China) were evaluated. The specimens were used with the written informed consent from the patient and the approval of the Ethics Committee of Southwest Hospital.

Immunohistochemistry was performed on 2 μm paraffin-embedded tissue sections using the avidin–biotin complex protocol. Briefly, to block endogenous peroxidase activity, all sections were treated with 0.3% (v/v) H_2_O_2_ at room temperature. Non-specific binding of possible endogenous biotin- or avidin-binding proteins was prevented through incubation with avidin/biotin blocking solutions. The primary anti-NUF2 antibody (1:200; Abcam, #ab122962) was applied to the sections after blocking with 10% normal goat serum. Next, biotin conjugated goat anti-rabbit IgG was applied to the sections as the secondary antibody and incubated. The slides were stained with DAB (3, 3′-diaminobenzidine; Sigma-Aldrich), and then dehydrated, cleared and mounted. Negative controls were performed by substitution of the primary antibody. NUF2 immunostaining photographs were acquired using a microscope (Leica, DMI4000B).

The slides were evaluated as described in the previous literature [20]. In brief, the level of NUF2 expression was scored according to the percentage of positively stained cells and the intensity of the colour, as follows: 0 (no positive cells), 1 (<1/3 positive cells), 2 (1/3–2/3 positive cells) and 3 (>2/3 positive cells); 0 (no colouration), 1 (pale yellow), 2 (yellow) and 3 (claybank). The two scores were combined to obtain the final one: 0, negative (−); 1–2, weakly positive (+); 3–4, moderately positive (++); 5–6; strongly positive (+++).

### Lentivirus construction and infection

The shRNA (small hairpin RNA) (5′-CCGGGAGAAATACC-ACGACGGTATTCTCGAGAATACCGTCGTGGTATTTCTC-TTTTTTG-3′) targeting human NUF2 gene (NM_031423) was designed and a scramble shRNA (5′-GCGGAGGG-TTTGAAAGAATATCTCGAGATATTCTTTCAAACCCTCC-GCTTTTTT-3′) was used as a negative control. Then they were ligated into lentiviral pFH-L plasmid (Shanghai Genechem). For lentivirus packaging, HEK-293T cells were transfected with pFH-L-NUF2 shRNA or control shRNA together with two helper plasmids (pVSVG-I and pCMVΔR8.92, Shanghai Genechem) using Lipofectamine™ 2000 (Invitrogen) as described in the manufacturer's instructions. Supernatant containing packaged lentivirus was collected and passed through 0.45 μm filters after 48 h of transfection. Then, lentivirus particles of shNUF2 (NUF2–siRNA) and shCon (scramble-siRNA) were added to the culture medium to infect human pancreatic cancer cell lines. After lentivirus infection, the cells were washed with PBS and collected to perform RT–PCR (reverse transcription–PCR) analysis and Western blot analysis.

### Real-time PCR analysis

Total mRNA was extracted from pancreatic cancer tissues and cultured cell lines using RNeasy Mini Kit (Qiagen). cDNA was then synthesized by RNA reverse transcribing with a Super Script III First-Strand Synthesis System for RT–PCR kit (Invitrogen). The expression level of NUF2 mRNA was measured by RT–PCR with an ABI PRISM 7000 Sequence Detection System (Applied Biosystems) with primers: 5′-TACCATTCAGCAATTTAGTTACT-3′ (forward); and 5′-TAGAATATCAGCAGTCTCAAAG-3′ (reverse). The primers of β-actin, used as internal control, were: 5′-CAGAGCCTCGCCTTTGCCGA-3′ (forward); and 5′-ACGCCCTGGTGCCTGGGGCG-3′ (reverse). Amplifications were then carried out and the PCR conditions were: initial denaturation at 95°C for 1 min, 40 cycles of denaturation at 95°C for 5 s and annealing extension at 60°C for 20 s. Relative quantification in RT–PCR was performed using 2^−ΔΔ^*C*_T_ (threshold cycle value) method [21]. Data were presented as *C*_T_ values, which were defined as the threshold PCR cycle number at which an amplified product is first detected. Δ*C*_T_=Avg. *C*_T_ (NUF2)–Avg. *C*_T_ (β-actin).

### Western blot analysis

Total proteins obtained from pancreatic cancer tissues and cultured cells were used for Western blot analysis. The protein concentration in cell extracts was measured using the BCA Protein Assay Kit (Beyotime). Equal amount of protein was loaded and separated by SDS–PAGE, and then transferred onto PVDF membranes (Millipore). The membrane was blocked with 5% (w/v) non-fat dried skimmed milk powder at room temperature, and incubated with primary antibody rabbit anti-NUF2 (1:1000; Abcam, #ab122962), rabbit anti-Cyclin B1 (1:1000; Abcam, #ab7957), rabbit anti-Cdc25A (1:1000; Abcam, #ab991), mouse anti-Cdc2 (1:1000; Cell Signaling, #9116), or rabbit anti-GAPDH (glyceraldehyde-3-phosphate dehydrogenase; 1:8000; Proteintech Group, Inc., #10494-1-AP). Then the membrane was washed and incubated with goat anti-rabbit HRP (horseradish peroxidase) secondary antibody (1:5000; Santa Cruz, #SC-2054) or goat anti-mouse HRP secondary antibody (1:5000; Santa Cruz, #SC-2005) as described in the manufacturer's instructions. Then the bands were visualized after incubation with chemiluminescence detection reagent (Pierce). The protein level of GAPDH was used as a loading control.

### Cell proliferation assay

To evaluate the effect of NUF2 knockdown on pancreatic cancer cell proliferation, MTT [3-(4,5-dimethylthiazol-2-yl)-2,5-diphenyl-2*H*-tetrazolium bromide] colorimetric assay was performed in both PANC-1 and Sw1990 cell lines *in vitro*. Briefly, 3 days after lentivirus infection, PANC-1 cells (2×10^3^/well) and Sw1990 cells (2.5×10^3^/well) were seeded into 96-well plates and incubated overnight at 37°C, respectively. Then 20 μl of MTT solution (5 mg/ml) was added to each well and incubated for 4 h. Then the medium was then removed, and 150 μl of DMSO was added to dissolve the formazan crystals. The absorption was measured at a wavelength of 590 nm. The measurements for each sample were conducted in triplicate.

### Colony formation assay

To examine the long-term effect of NUF2 knockdown on pancreatic cancer cell proliferation, colony formation assay was performed in PANC-1 cells. Briefly, 3 days after lentivirus infection, about 400 PANC-1 cells were seeded in 6-well plates (Corning). Cells were cultured at 37°C for 10 days to allow colony formation. Cells were then washed by PBS and fixed with 4% PFA (paraformaldehyde) and stained with 0.1% crystal violet (Sigma-Aldrich). Then images were captured by a fluorescence microscope (Leica). The number of colonies (>50 cells/colony) was counted.

### Cell cycle analysis

The effect of NUF2 knockdown on cell cycle progression of pancreatic cancer cells was determined by flow cytometry with propidium iodide staining. Briefly, 3 days after lentivirus infection, PANC-1 cells (3×10^4^/well) and Sw1990 cells (3.5×10^4^/well) were seeded into 6-well plates and incubated at 37°C for 40 h. Then cells were harvested, fixed in 70% (v/v) ethanol, and stored overnight at 4°C. The cells were resuspended in cold PBS and incubated in a solution containing 10 mg/ml RNase and 1 mg/ml propidium iodide (Sigma-Aldrich). Following incubation for 1 h in the dark at room temperature, cells were measured by flow cytometry (FACS Calibur, BD Biosciences). The percentage of cells in different phases of the cell cycle was determined.

### *In vivo* experiment

Male BALB/c nude mice of 5 weeks of age (*n*=12) were obtained from Third Military Medical University (Chongqin, China) and kept under SPF (specific pathogen-free) conditions. All animal experiments were evaluated and approved by the Ethics Committee of Southwest Hospital.

PANC-1 cells were previously infected with shNUF2 and shCon for 96 h. Then each nude mouse was injected subcutaneously in the right flank with the treated PANC-1 cells (5×10^6^/site) to establish xenograft nude mouse models of pancreatic cancer. Then the tumour volumes were measured every 3–4 days with a micrometer calliper using the formula: tumour volume (mm^3^)=1/2 (a×b^2^), where a is the longest longitudinal diameter and b is the longest transverse diameter. Tumour growth was followed for 28 days from the first injection. Then the mice were killed by cervical and the tumours were then excised to measure the weights and conduct PCNA (proliferating cell nuclear antigen) immunofluorescence assay.

### Immunofluorescence staining

The expression of PCNA was detected by immunofluorescence. Deparaffinized 4-μm tissue sections were cultured with primary antibody mouse anti-PCNA (1:800; Abcam, #ab29). Subsequent antibody detection was carried out with Alexa Fluor 488 goat anti-mouse IgG (1:500; Invitrogen) secondary antibody. Sections were examined with a fluorescence microscope, and merged images were formed using Adobe Photoshop CS4.

### Statistical analysis

Statistical analyses were performed with SPSS 13.0 software. The results of immunohistochemistry were evaluated by χ^2^ test and the other data were evaluated by Student's *t* test and expressed as the means±S.D. from three independent experiments. A *P*-value of less than 0.05 was considered statistically significant.

## RESULTS

### NUF2 was associated with pancreatic cancer progression

The expression of NUF2 was evaluated in 128 PDAC specimens by immunohistochemical staining. NUF2 expression was positive in more than 90% of PDAC tissues. Representative photographs of immunohistochemical staining are shown in Figure 1. Compared with normal adjacent tissue, NUF2 was intensely stained in PDAC tissues. Moreover, higher expression of NUF2 was found to be significantly associated with lymph node metastasis (*P*=0.036) and higher TNM stage (*P*=0.003) (χ^2^ test, Table 1). It is reasonable to assume that the overexpression of NUF2 may be associated with poor prognosis for patients with pancreatic cancer.

**Figure 1:** Immunohistochemical analysis of NUF2 expression in human PDAC specimens Positive cells were stained brown. (**A**) NUF2-negative staining in normal adjacent tissue. (**B**, **C**) NUF2-positive staining in PDAC tissues. Scale bars=50 μm.

**Table 1:** Relationship of NUF2 expression and clinicopathological parameters in PDAC patients (*n*=128) *P* values were determined using a Pearson χ^2^ test.

		NUF2 immunostaining		
Characteristic	*n*	-/+	++/+++	*P*
Age				
≤62 years	65	29	36	0.263
>62 years	63	22	41	
Gender				
Female	59	19	40	0.103
Male	69	32	37	
Tumour location				
Head	56	20	36	0.400
Body/tail	72	31	41	
Tumour size				
≤2 cm	29	10	19	0.445
2–4 cm	57	21	36	
>4 cm	42	20	22	
Lymph node metastasis				
N0	84	39	45	0.036*
N1	44	12	32	
Tumour differentiation				
Well/moderate	89	37	52	0.546
Poor	39	14	25	
TNM stage				
I/II	95	45	50	0.003**
III/IV	33	6	27	

### NUF2 was highly expressed in pancreatic cancer tissues and cell lines

To evaluate the functional role of NUF2 in pancreatic cancer, the expression levels of NUF2 were examined in 15 cases of pancreatic cancer tissues and four human pancreatic cancer cell lines, including Sw1990, PANC-1, BXPC-3, and MLA-PACA-2, as well as the HEK-293 cells. As shown in Figure 2(A), NUF2 mRNA levels in pancreatic cancer tissues were nearly 3.3-fold increased relative to those in adjacent non-cancerous tissues. In addition, NUF2 mRNA was highly expressed in a set of human pancreatic cancer cell lines, rather than HEK-293 cell line (Figure 2B). Higher protein levels of NUF2 were also observed in pancreatic cancer cell lines relative to HEK-293 cell line (Figures 2C and 2D). These results indicated that NUF2 is significantly elevated in pancreatic cancer tissues and cell lines. Importantly, PANC-1 cell line showed the highest NUF2 expression, and thus was selected as an optimal cell model along with Sw1990 cell line for our subsequent loss-of-function experiments.

**Figure 2:** NUF2 expression in human pancreatic cancer tissues and cell lines (**A**) RT–PCR analysis of NUF2 expression in 15 pairs of pancreatic cancer and normal adjacent tissues. **P<0.01, compared with normal tissues. (**B**) RT–PCR analysis of NUF2 expression in four human pancreatic cancer cell lines and HEK-293 cell line. β-actin gene was used as an internal gene. Data represent the means±S.D. of three independent experiments. *P<0.05, **P<0.01, compared with HEK-293 cells. (**C**, **D**) Western blot analysis of NUF2 expression in four human pancreatic cancer cell lines and HEK-293 cell line. GAPDH protein was used as an internal control. Data represent one of the three independent experiments with similar results. *P<0.05, **P<0.01, compared with HEK-293 cells.

### lentivirus-mediated siRNA decreased endogenous NUF2 expression in pancreatic cancer cells

To evaluate the physiological function of NUF2 in pancreatic cancer cells, we employed lentivirus-mediated siRNA to knock down NUF2 expression in PANC-1 and Sw1990 cells. As shown in Figures 3(A) and 3(B), compared with un-infected (Con) and shCon-treated groups, the mRNA levels of NUF2 in shNUF2 groups were dramatically reduced in both PANC-1 and Sw1990 cell lines. However, there was no difference between the shCon-treated group and Con group. Western blot analysis also verified the down-regulation of NUF2 expression in both cell lines at protein levels (Figures 3C and 3D). These results indicated that lentivirus-mediated siRNA was able to specifically knock down endogenous NUF2 expression in pancreatic cancer cells.

**Figure 3:** Knockdown efficiency of lentivirus-mediated siRNA targeting NUF2 in pancreatic cancer cells RT–PCR analysis of NUF2 knockdown efficiency in PANC-1 cells (**A**) and Sw1990 cells (**B**), respectively. β-actin gene was used as an internal gene. Data represent the means±S.D. of three independent experiments. **P<0.01, ***P<0.001, compared with shCon. Western blot analysis of NUF2 knockdown efficiency in PANC-1 cells (**C**) and Sw1990 cells (**D**), respectively. GAPDH protein was used as an internal control. Data represent one of the three independent experiments with similar results.

### NUF2 knockdown decreased proliferation and colony formation of pancreatic cancer cells

To explore the functional role of NUF2 in pancreatic cancer cell growth, MTT assay was firstly performed in PANC-1 and Sw1990 cells. As shown in Figure 4(A), the proliferative rate of PANC-1 cells was remarkably reduced after shNUF2 infection, compared with Con and shCon-treated groups. The difference concerning cell viability reached to peak on day 5 (*P*<0.001). Similarly, the proliferative rate of Sw1990 cells was also decreased by NUF2 knockdown (*P*<0.01, Figure 4B). These results indicated that silencing of NUF2 could potently suppress proliferation of pancreatic cancer cells.

**Figure 4:** Effects of NUF2 knockdown on proliferation and colony formation of pancreatic cancer cells Growth curves of PANC-1 cells (**A**) and Sw1990 cells (**B**) with three treatments (Con, shCon and shNUF2) determined by MTT assay. Data represent the means±S.D. of three independent experiments. **P<0.01, ***P<0.001, compared with shCon. (**C**) Representative images recorded under micro and macro view, representing the size and the number of colonies in each group of cells. Scale bars=250 μm. (**D**) Colony numbers of PANC-1 cells were counted. Data represent the means±S.D. of three independent experiments. ***P<0.001, compared with shCon.

Next, we conducted colony formation assay to evaluate long-term cell proliferation capacity. Crystal violet staining and fluorescence expression showed that both the size of monoclone and the number of total colonies were decreased in shNUF2-treated groups, compared with Con and shCon-treated groups (Figure 4C). The colony formation ability was visibly impaired in PANC-1 cells after NUF2 knockdown. As shown in Figure 4(D), the colony numbers of the shNUF2-treated group (28.7±6.8) were significantly fewer than those of shCon-treated (165.0±12.5) and Con (153.0±13.7) groups. It could be concluded that silencing of NUF2 could disrupt the tumourigenicity of pancreatic cancer cells *in vitro*.

### NUF2 knockdown blocked cell cycle progression of pancreatic cancer cells

To evaluate the mechanism underlying shNUF2-mediated cell growth inhibition, the cell cycle distribution in both PANC-1 and Sw1990 cell lines was detected by flow cytometry (Figures 5A and 5C). As shown in Figure 5(B), when NUF2 expression was silenced, the cell cycle progression of PANC-1 cells was blocked, with a remarkable increase in the percentage of cells in the G0/G1 phase (83.94±1.56% in the shNUF2-treated group versus 71.86±2.86% and 73.09±3.65% in shCon-treated and Con groups, *P*<0.05); in addition, a significant decrease in cell percentage of S phase (7.75±1.69% versus 12.52±0.25% and 12.57±1.65%, *P*<0.05) and G2/M phase (8.31±0.95% versus 15.62±1.25% and 14.34±1.25%, *P*<0.05). Similarly, NUF2 knockdown in Sw1990 cells also resulted in a significant increase of cell percentage in the G0/G1 phase and a concomitant decrease in cell population of G2/M phase (Figure 5D). These results indicated that silencing of NUF2 by siRNA in pancreatic cancer cells could induce cell cycle arrest at G0/G1 phase.

**Figure 5:** Effect of NUF2 knockdown on cell cycle progression pancreatic cancer cells Cell cycle distribution of PANC-1 cells (**A**) and Sw1990 cells (**C**) with three treatments (Con, shCon and shNUF2) determined by flow cytometric analysis. (**B**, **D**) The percentage of cells in the G0/G1, S and G2/M phases of the cell cycle was counted. Data represent the means±S.D. of three independent experiments. *P<0.05, **P<0.01, compared with shCon.

### NUF2 knockdown down-regulated cell cycle regulators

To further confirm the molecular basis for NUF2-mediated cell cycle progression, we evaluated the expression alterations of cell-cycle-related proteins in both PANC-1 and Sw1990 cell lines. As shown in Figures 6(A) and 6(B), the cell cycle key mediators G2/M phase-related Cyclin B1, Cdc25A and Cdc2 were all down-regulated in response to NUF2 inhibition, which suggested that NUF2 knockdown probably blocked cell cycle progression through down-regulation of Cyclin B1, Cdc25A and Cdc2.

**Figure 6:** Knockdown of NUF2 down-regulated cell cycle regulators in pancreatic cancer cells Western blot analysis of Cyclin B1, Cdc25A and Cdc2 expression in PANC-1 cells (**A**) and Sw1990 cells (**B**) after NUF2 knockdown. Data represent one of the three independent experiments with similar results.

### NUF2 knockdown inhibited the tumour growth *in vivo*

The human xenograft nude mouse models of pancreatic cancer were successfully developed using shNUF2-treated or shCon-treated PANC-1 cells. As the time of implantation prolonged, the tumour volume in each group showed a progressive increase, but the growth rate in the shNUF2 group was significantly slower than in the shCon group. After 27 days of implantation, the mean tumour volume was dramatically smaller in the shNUF2-treated group (242±60 mm^3^) than in the shCon-treated group (523±80 mm^3^) (*P*<0.05, Figure 7A). Moreover, compared with the shCon-treated group, the tumour weight in the shNUF2-treated group was also significantly decreased (*P*<0.05, Figure 7B). Representative images of solid tumours are shown in Figure 7(C). Immunohistochemical staining of NUF2 further verified that its expression was obviously reduced in tumour tissues after shNUF2 treatment (Figure 7D).

**Figure 7:** Knockdown of NUF2 inhibited tumour growth in pancreatic cancer xenograft nude mice (**A**) Growth curves of xenograft tumours in nude mouse models. (**B**) Weight of xenograft tumours in nude mouse models. (**C**) Representative images recorded under macro view, representing the size of tumours in nude mice. Data represent the means±S.D. from six nude mouse models. (**D**) Immunohistochemical analysis of NUF2 expression in tumours after shNUF2 treatment. Positive cells were stained brown. Scale bars=50 μm.

We further investigated whether NUF2 could modulate the expression of the proliferation biomarker PCNA in tumour tissues. Through immunofluorescent staining, we observed that the expression of PCNA was remarkably reduced in the shNUF2 group than in the shCon group (Figure 8), which could contribute to a decreased proliferative activity of cancer cells induced by NUF2 knockdown. Taken together, our data demonstrated that NUF2 knockdown was able to inhibit the proliferation of pancreatic cancer cells *in vivo*, thus suppress *in vivo* tumourigenesis in pancreatic cancer xenograft nude mice.

**Figure 8:** Immunofluorescent images illustrate location of PCNA protein in tumour tissue of pancreatic cancer nude mice Green fluorescence shows nuclear expression of PCNA, and blue fluorescence shows all cell nuclei with patterns of DAPI (4′,6-diamidino-2-phenylindole) staining. Data represent one of the three independent experiments with similar results. Scale bars=50 μm.

## DISCUSSION

The highly conserved Ndc80–NUF2 complex is involved in kinetochore interactions and the spindle assembly checkpoint in mitosis [18]. Among the Ndc80–NUF2 complex, NUF2 is required for kinetochore integrity and the organization of stable microtubule-binding sites in the outer plate of the kinetochore [11]. As we know, mitosis dysregulation is a common cause in carcinogenesis [22,23]. In previous studies, the Ndc80–NUF2 complex has been reported to be implicated in the development of multiple human cancers [13–18]. In the present study, we primarily found that NUF2 was expressed in 90% of PDAC specimens collected from 128 patients. Moreover, higher NUF2 expression was positively associated with worse clinicopathological variables, including lymph node metastasis and higher TNM stage, which predicts poor prognosis in pancreatic cancer. NUF2 was also aberrantly overexpressed in pancreatic cancer tissues and cell lines, implying the involvement of NUF2 in pancreatic cancer.

To examine the biological role of NUF2 in pancreatic cancer cell growth, we conducted loss-of-function analysis using lentivirus-mediated siRNA in PANC-1 and Sw1990 cells. Silencing of NUF2 significantly inhibited the proliferation and colony formation ability of pancreatic cancer cells *in vitro* through inducing cell cycle arrest at G0/G1 phase. Cyclin B1 and Cdc2 are key molecules for G2–M transition during the cell cycle. Cyclin B1 is essential for the initiation of mitosis and suppression of Cyclin B1 could lead to cells block and eventual cell apoptosis [24]. Similarly, after the down-regulation of Cdc25A, cell cycle progression was inhibited [25,26]. In this study, the expression levels of Cyclin B1, Cdc25A and Cdc2 were all decreased in both PANC-1 and Sw1990 cell lines after NUF2 silencing, which could contribute to cell cycle arrest and eventual cell growth inhibition.

Additionally, siRNA-based drugs have also proven to be feasible options for *in vivo* therapy [27,28]. Therefore, we further measured the effectiveness of targeting NUF2 using xenograft mouse models of pancreatic cancer. It is noteworthy that NUF2 knockdown markedly inhibited the growth of xenografts in nude mice. Taken together, depletion of NUF2 by siRNA could remarkably inhibit pancreatic cancer growth both *in vitro* and *in vivo*. PCNA is a nuclear protein associated with the cell cycle whose immunolocalization can be used as a marker to study cell proliferation. There is a clear correlation between up-regulation of PCNA expression and increased cell proliferation [29,30]. Furthermore, immunofluorescent staining of PCNA showed that its expression was visibly reduced in tumour tissues after shNUF2 treatment, which suggested that the elevated PCNA expression could participate in NUF2-induced pancreatic tumourigenesis *in vivo*.

In fact, kinetochore components, particularly NDC80 and NUF2, have already been proposed as potential targets for cancer therapeutics [14]. Thus, we suggest that NUF2 may be a promising biomarker in pancreatic cancer that can provide information not only for predicting disease occurrence, but also suggesting treatment options, which can be personalized to the patient. Currently, the most promising inhibitor targeting the NDC80/NUF2 pathway is INH11, which disrupts the formation of Ndc80–NUF2 complex, has been shown to reduce proliferation in breast cancer cells and reduce tumour growth in a xenograft mouse model [31]. Therefore the small molecular inhibitor INH11 targeting NUF2 could potentially be used as a novel therapy for pancreatic cancer. Functional analyses of NUF2 depletion in pancreatic cancer cells via INH11 are required for further validation of our results.

In conclusion, we provide new evidence that NUF2 is closely linked with pancreatic cancer development and progression. Our study represents the first report on NUF2 as a potential drug target for treatment of pancreatic cancer.
